This article has been retracted.

# Effects of Different Nonsteroidal Anti-Inflammatory Drugs Combined with Platelet-Rich Plasma on Inflammatory Factor Levels in Patients with Osteoarthritis

**DOI:** 10.1155/2022/1979892

**Published:** 2022-03-31

**Authors:** Wenxiao Jiang, Yijun Zhang, Ye Huang, Yunfeng Cheng

**Affiliations:** ^1^Department of Sports Medicine, Qilu Hospital of Shandong University, Qingdao 266035, Shandong, China; ^2^Department of Surgery of Traditional Chinese Medicine, The People's Hospital of South District of Qingdao, Qingdao 266000, Shandong, China; ^3^Department of Orthopedic Surgery, Haiyang Chinese Medicine Hospital, Yantai 265100, Shandong, China

## Abstract

**Objective:**

To investigate the effects of different nonsteroidal anti-inflammatory drugs combined with platelet-rich plasma on inflammatory factor levels in patients with osteoarthritis.

**Methods:**

The clinic data of 120 patients with osteoarthritis who were treated in our hospital (June 2019-June 2021) were retrospectively reviewed. All the patients were given platelet-rich plasma. According to the different nonsteroidal anti-inflammatory drugs the patients received, they were equalized into diclofenac sodium group, celecoxib group, and iguratimod group, with 40 cases in each group. After treatment, the patients' clinical efficacy was compared and analyzed.

**Results:**

After treatment, the pain degrees of the patients in the three groups were gradually reduced. After 4 weeks and 8 weeks of treatment, the statistical differences in the scores of Visual Analogue Scale (VAS) were found among the three groups. Specifically, compared with the other two groups, the iguratimod group had remarkably lower VAS scores (*P* < 0.05) and the celecoxib group had signally lower VAS scores compared with the diclofenac sodium group (*P* < 0.05). After treatment, the inflammatory factor levels of interleukin-6 (IL-6), tumor necrosis factor-*α* (TNF-*α*), and high-sensitivity C-reactive protein (hs-CRP) in the diclofenac sodium group were observably higher compared with the celecoxib group (*P* < 0.05), and the inflammatory factor levels in the celecoxib group were remarkably higher compared with the iguratimod group (*P* < 0.05). Before treatment, no notable difference in the Lysholm scores was found among the three groups, and the patients' knee joint function was gradually improved after treatment. To be specific, after 4 and 8 weeks of treatment, the iguratimod group had observably higher Lysholm scores compared with the other two groups (*P* < 0.05), and the celecoxib group had signally higher Lysholm scores compared with the diclofenac sodium group (*P* < 0.05). The iguratimod group got markedly lower Western Ontario and McMaster Universities (WOMAC) score compared with the celecoxib group (*P* < 0.05); Compared with the diclofenac sodium group, the celecoxib group got remarkably lower WOMAC score (*P* < 0.05). During treatment, few patients suffered from mild gastrointestinal discomfort and hepatic dysfunction in the three groups, and no other severe adverse reactions were found. No statistical difference in the total incidence of adverse reactions among the three groups was observed (*P* > 0.05).

**Conclusion:**

The combination of nonsteroidal anti-inflammatory drugs with platelet-rich plasma can further reduce the inflammatory reactions of the patients with osteoarthritis and improve their knee joint function. Significantly, the iguratimod, with high safety, has observably better effects on inhibiting inflammatory factors and improving knee joint function compared with diclofenac sodium and celecoxib.

## 1. Introduction

Osteoarthritis, as a chronic disease, mainly damages the articular cartilage, with pain, stiffness, and limited movement as the main clinical symptoms. The principle of treating osteoarthritis in clinic is providing graded and individualized treatment according to the patients' conditions. Especially for the patients in early or medium stage, the stage treatment measures should be improved as much as possible, which is the current research hotspot in this field. Platelet-rich plasma is the platelet concentration made by the isolated autologous whole blood, and includes a great deal of growth factors and proteins. Platelet-rich plasma can repair damaged cartilage and promote bone healing and has been widely used in orthopedics in recent years. Many previous clinical trials have shown that injecting the platelet-rich plasma into the articular cavity can relieve clinical symptoms of patients with mild and moderate osteoarthritis with effect and can significantly inhibit the expression of inflammatory factors and the degradation of cartilage matrix [1–4]. In the clinical treatment of osteoarthritis, the platelet-rich plasma is frequently adopted in combination with other methods. In addition, when the basic treatment for osteoarthritis is ineffective, the nonsteroidal anti-inflammatory drugs (NSAIDs) are the first choice in further treatment. Besides, they are also the most commonly used drugs to relieve pain and improve joint function in patients with osteoarthritis. The combination of NSAIDs and platelet-rich plasma can guarantee the clinical efficacy of the patients with osteoarthritis. However, it has been found that different NSAIDs can cause different degrees of rash, renal impairment, gastrointestinal complications, and cardiovascular and cerebrovascular risks in the clinical course of medication[5–8]. Based on previous studies, this paper further investigates the effects of different NSAIDs (diclofenac sodium, celecoxib, and iguratimod) combined with platelet-rich plasma on inflammatory factor levels in patients with osteoarthritis.

## 2. Materials and Methods

### 2.1. Patients Screening

Inclusion criteria were as follows: ① The patients matched the diagnostic standards for osteoarthritis in Guideline for Clinical Diagnosis and Treatment of Osteoarthritis (2021) [9], and their diagnoses were confirmed by imaging examinations; ② the patients 50 years old or older; ③ the patients' synovial fluid was yellow, with positive coagulation test, and the leucocyte count in synovial fluid was lower than 2 × 106/L; ④ the patients' clinical data were complete; and ⑤ the patients and their families were informed of the study and had signed the informed consent. Exclusion criteria were as follows: ① the patients suffered from severe joint deformity; ② the patients were complicated with immune dysfunction, coagulation disorders, organic diseases, or malignant tumors; ③ the patients had bacterial arthritis, gouty arthritis, rheumatoid arthritis, or other joint diseases; ④ the patients had the illness history of ligament rupture or meniscus injury; ⑤ the patients had received surgery on the knees; ⑥ the patients had cognition disorders, language dysfunction or audio-visual disorders; and ⑦ the patients' conditions were extremely unstable. In the light of the above criteria, 120 patients with osteoarthritis who were treated in our hospital (June 2019–June 2021) were chosen as the study objects.

### 2.2. Grouping

According to the different nonsteroidal anti-inflammatory drugs the patients received, they were equalized into diclofenac sodium group, celecoxib group, and iguratimod group, and each group had 40 patients. The Hospital Ethics Committee approved this study and was conducted under supervision of this Committee.

### 2.3. Methods

After the acute stage treatment, the patients in the three groups received different nonsteroidal anti-inflammatory drugs. Patients from the diclofenac sodium group orally took diclofenac sodium sustained release tablets (Specification: 0.1 g; Manufacturer: Sinopharm Zhijun (Shenzhen) Pingshan Pharmaceutical Co., Ltd; NMPA Approval No. H10970209), once a day and 1 tablet once. The patients in the celecoxib group orally took celecoxib capsules (Specification: 0.2 g; Manufacturer: Pfizer Pharmaceuticals LLC; NMPA Approval No. J20120063), once a day and 1 tablet once. The patients in the iguratimod group orally took iguratimod tablets (Specification: 25 mg; Manufacturer: Simcere Pharmaceutical Group Limited; NMPA Approval No. H20110084) after meals in the morning and evening, twice a day and 1 tablet once.

Platelet-rich plasma: all the patients received the treatment of platelet-rich plasma. Forty milliliters of the blood from antecubital vein was collected and the platelet-rich plasma was made by the two-step centrifugation method. The blood was centrifuged at 1450 r/min for 10 minutes for first time. Then, all the clear supernatant and the solid between the solid-liquid interface and 3 mm below the interface were collected and centrifuged at 3370 r/min for 10 minutes. After that, 3/4 of the clear supernatant was removed and the rest was the platelet-rich plasma [10, 11]. Four milliliters of the platelet-rich plasma was injected into the joint lesion sites, and 1 ml of calcium chloride was added to the plasma before injection to activate the platelets. The patients received such treatment once a week, and one course of treatment lasted for three weeks. The patients received two courses, with 1-week interval between the two courses.

### 2.4. Observed Indexes

The patients' age, course of disease, body mass index (BMI), sex, focus of infection, K-L classification, educational level, and other general data were collected. Besides, 5 ml of fasting venous blood was drawn and collected, with serum being separated from the blood sample. Then, the patients' inflammatory factor levels of interleukin-6 (IL-6) and tumor necrosis factor-*α* (TNF-*α*) was determined by enzyme-linked immunosorbent assay. Their high-sensitivity C-reactive protein (hs-CRP) levels were determined by immunoturbidimetry.

Severity of pain: the Visual Analogue Scale (VAS), with high sensitivity, was adopted to evaluate the patients' severity of pain. The patients needed to look at the “pain scale” (a 10-centimeter-long vernier caliper, with 10 scales marked on one side and “0” and “10” at both ends) and to state a number between 0 and 10. Zero signified no pain; 1–3 points signified slight pain which was tolerable; 4–6 points signified the tolerable pain which influenced the patients' sleep; 7–9 points signified the intolerable pain which became gradually intense and influenced the patients' sleep and appetite; and 10 points represented the intolerable severe pain.

Knee joint function: the Lysholm knee scoring scale [12] was employed to assess patients' knee joint function. This scale was formulated by Lysholm and Gillquist in 1982, and its validity and reliability have been confirmed by clinical trials. This scale included 8 items of limp, support, locking, pain, instability, swelling, stair climbing, and squatting, with the total score of 100 points. Higher points indicated better knee joint function.

Osteoarthritis index: The Western Ontario and McMaster Universities (WOMAC) Osteoarthritis Index was employed to assess the severity of osteoarthritis and clinical efficacy and included three aspects of pain, stiffness and physical function, with 24 items in total. This scale covered the basic symptoms and physical signs of osteoarthritis, and higher scores indicated more severe osteoarthritis. The Cronbach's *α* coefficients of every dimension was 0.6–0.83, and factor analysis showed good construct validity.

The patients' adverse reactions during treatment were recorded and collected.

### 2.5. Statistical Treatment

In this study, the software SPSS22.0 was adopted to calculate the differences among groups and GraphPad Prism 7 (GraphPad Software, San Diego, USA) was used to draw graphs of the data. The study included count data and measurement data. The count data were tested by X^2^ and expressed by (*n* (%)). The measurement data were tested by *t* and expressed by (‾*x* ± *s*). When *P* < 0.05, the differences were considered statistically significant.

## 3. Results

### 3.1. General Data

No notable difference in age, course of disease, body mass index (BMI), sex, focus of infection, K-L classification, educational level, and other general data was discovered among the three groups (*P* > 0.05; Table 1).

Grade I: the joint space was suspected of becoming narrow, and the osteophyte might occur; Grade II. the patients had obvious osteophyte, and the joint space was suspected of becoming narrow.

From the perspective of the severity of knee osteoarthritis, the patients in grade I and grade II accorded with the study object.

### 3.2. Severity of Pain

The pain degrees of the patients in the three groups were gradually reduced after treatment. After 4 weeks and 8 weeks of treatment, the statistical differences in the VAS scores were found among the three groups. Specifically, the iguratimod group had remarkably lower VAS scores compared with the other two groups (*P* < 0.05), and the celecoxib group had signally lower VAS scores compared with the diclofenac sodium group (*P* < 0.05; Figure 1).

### 3.3. Inflammatory Factor Levels

According to the statistical data in Table 2, IL-6, TNF-*α*, and hs-CRP in the diclofenac sodium group were observably higher compared with the celecoxib group after treatment (*P* < 0.05). The celecoxib group achieved remarkably higher inflammatory factor levels compared with the iguratimod group after treatment (*P* < 0.05).

### 3.4. Knee Joint Function

Before treatment, no notable difference in the Lysholm scores was found among the three groups, and the patients' knee joint function was gradually improved after treatment. To be specific, after 4 weeks and 8 weeks of treatment, the iguratimod group had observably higher Lysholm scores compared with the other two groups (*P* < 0.05), and the celecoxib group had signally higher Lysholm scores compared with the diclofenac sodium group (*P* < 0.05; Table 3).

### 3.5. Osteoarthritis Indexes

The iguratimod group got markedly lower WOMAC score compared with the celecoxib group (*P* < 0.05). Compared with the diclofenac sodium group, the celecoxib group got remarkably lower WOMAC score (*P* < 0.05; Figure 2).

### 3.6. Adverse Reactions

During treatment, there were few cases suffering from mild gastrointestinal discomfort and hepatic dysfunction in the three groups, and no other severe adverse reactions were found. No statistical difference in the total incidence of adverse reactions among the three groups was discovered (*P* > 0.05).

## 4. Discussion

Osteoarthritis is a progressive joint disease induced by the imbalance of intra-articular stress function and characterized by the repair disorders of articular cartilages. The main physiological changes are progressive destruction of the affected articular cartilage and imbalance between the articular cartilage's decomposition and anabolism, and the synthesis and decomposition caused by dysregulation of various cytokines play an important role in joint degeneration [13]. Therefore, how to repair damaged cartilage and prevent further damage is the key to treating osteoarthritis. At the same time, understanding the damage mechanism of articular cartilage tissue is a prerequisite for the treatment of osteoarthritis. According to modern basic medical research, polypeptide growth factors can regulate the synthetic and catabolic processes of cartilage [14]. Under normal circumstances, the balance between synthesis and decomposition of articular cartilage matrix is maintained by the dynamic balance in quantity between the synthetic and catabolic cytokines in the body. IL-6 and TNF-*α* are the important catabolic cytokines involved in the pathogenesis of osteoarthritis and are closely related to the degradation of intra-articular cartilage matrix, synovial lesion and reduction of chondrocyte function in patients with osteoarthritis. After the extracellular matrix of articular cartilage is decomposed by a variety of MMPs, the articular cartilage expands. As a result, the resistance of articular cartilage to the outside world is reduced, causing further damage to the articular cartilage. Generally, there is little differences in the amount between synthetic cytokines and catabolic cytokines in the early stage of osteoarthritis. The disease progression caused by untimely treatment leads to the degeneration of more articular chondrocytes, and the production of plentiful catabolic cytokines, like the overexpression of IL-6, TNF-*α*, hs-CRP, and so on. As a result, the chondrocytes are inhibited from dividing and the proteoglycan is inhibited from synthesizing. With the pathological increase of catabolic cytokines, the inflammatory factors of IL-6, TNF-*α,* and hs-CRP trigger immune response and aggravate cartilage injury.

Platelet-rich plasma, the plasma whose platelet concentration is 2–7 times the concentration of the whole blood, has been widely employed in bone and joint diseases at present. Meanwhile, the treatment of osteoarthritis is also one of the important research directions. In the treatment of osteoarthritis, platelet-rich plasma has the advantages of minimal invasion, economy, less complications, and less pain compared with surgical treatment [15, 16]. Platelet-rich plasma, rich in various growth factors and cytokines, plays a crucial part in the normal expression of cartilage cells and is an important treatment measure to regulate the dynamic balance between synthetic cytokines and catabolic cytokines. In addition, NSAIDs are also commonly used in the early treatment of osteoarthritis, and their mechanisms of action are as follows: (1) NSAIDs reduce the synthesis of prostaglandin by inhibiting cyclooxygenase activity; (2) NSAIDs can reduce the stimulation to nerve endings by inhibiting lymphocyte activity and differentiation of activated T lymphocytes; and (3) NSAIDs act directly on polymodal nociceptors to block the formation and release of pain-producing substances [17–20]. Cyclooxygenase includes two isozymes—cyclooxygenase-1 (COX-1) and cyclooxygenase-2 (COX-2). COX-1, a kind of constitutive enzyme, mostly exists in gastrointestinal tract and kidney and can promote the synthesis of physiological prostaglandins and regulate the physiological activities of normal tissue cells. COX-2, an inducible type enzyme, is generated under the induction of injury or inflammatory factors and catalyzes the synthesis of prostaglandins, triggering a series of inflammatory responses and pain. According to previous studies, while relieving the patients' postoperative pain, NSAIDs could also inhibit the release of bradykinin and exert anti-inflammatory effect by controlling the platelet concentration [21–24].

In this study, all the patients received different NSAIDs (diclofenac sodium, celecoxib, and iguratimod) combined with platelet-rich plasma and the patients' clinic data were retrospectively reviewed. The treatment results were as follows. The pain degrees of the patients in the three groups were gradually reduced after treatment. After 4 weeks and 8 weeks of treatment, the statistical differences in the VAS scores were found among the three groups. Specifically, compared with the other two groups, the iguratimod group had remarkably lower VAS scores (*P* < 0.05); compared with the diclofenac sodium group, the celecoxib group had signally lower VAS scores (*P* < 0.05). These results were in line with the research report of PU CHUNXUE et al. [25], confirming that all the NSAIDs had good analgesic effects and iguratimod had a better analgesic effect compared with the other two drugs. After treatment, the inflammatory factor levels of IL-6, TNF-*α*, and hs-CRP in the diclofenac sodium group were observably higher compared with the celecoxib group (*P* < 0.05), and the inflammatory factor levels in the celecoxib group were remarkably higher compared with the iguratimod group (*P* < 0.05). Before treatment, no notable difference in the Lysholm scores was discovered among the three groups, and the patients' knee joint function was gradually improved after treatment. To be specific, after 4 and 8 weeks of treatment, the iguratimod group had observably higher Lysholm scores compared with the other two groups (*P* < 0.05), and the celecoxib group had signally higher Lysholm scores compared with the diclofenac sodium group (*P* < 0.05). The iguratimod group got markedly lower WOMAC score compared with the celecoxib group (*P* < 0.05). Compared with the diclofenac sodium group, the celecoxib group got remarkably lower WOMAC score (*P* < 0.05). According to these results, iguratimod had better anti-inflammatory effect and better improvement of knee joint function in patients with osteoarthritis compared with celecoxib and diclofenac sodium, and the efficacy of celecoxib was better than that of diclofenac sodium. Diclofenac sodium, as a kind of nonspecific NSAIDs, inhibits the inflammatory response and relieves pain by promoting the synthesis of proteoglycans in the cartilage matrix. Diclofenac sodium exerts the inhibition of both COX-1 and COX-2. Celecoxib, as a kind of specific NSAIDs, only inhibits COX-2. Iguratimod, a kind of new NSAIDs, can exert anti-inflammatory effects by inhibiting the bradykinin in inflammatory response and inhibit the immunoglobulins of B cells from generating. Iguratimod can also control rheumatoid arthritis (RA) and bone loss caused by RA by inhibiting IL-1*β*, TNF-*α*, IL-6, IL-8, MPC-1, and other cytokines from synthesizing, so as to prevent bone absorption and promote bone formation. During treatment, there were few cases suffering from mild gastrointestinal discomfort and hepatic dysfunction in the three groups, and no other severe adverse reactions were found. No statistical difference in the total incidence of adverse reactions among the three groups was discovered (*P* > 0.05), which might be caused by the small sample size, and the sample size should be enlarged in the follow-up studies.

In conclusion, the combination of NSAIDs with platelet-rich plasma can further reduce the inflammatory reactions of the patients with osteoarthritis and improve their knee joint function. Significantly, iguratimod, with high safety, has observably better effects on inhibiting inflammatory factors and improving knee joint function compared with diclofenac sodium and celecoxib. Therefore, the iguratimod is the first choice in clinic and can be used in combination with the other two drugs according to the patients' conditions, but its dosage should be paid attention to.

## Figures and Tables

**Figure 1:** Comparison of VAS scores. The abscissa indicated before treatment, after 4 weeks of treatment, and after 8 weeks of treatment, and the ordinate indicated the VAS score (points). The VAS scores in the diclofenac sodium group before treatment, after 4 weeks of treatment, and after 8 weeks of treatment were (6.33 ± 1.42), (5.64 ± 1.06), and (4.01 ± 0.58) points, respectively. The VAS scores in the celecoxib group before treatment, after 4 weeks of treatment, and after 8 weeks of treatment were (6.35 ± 1.35), (4.59 ± 1.02), and (3.50 ± 0.82) points, respectively. The VAS scores in the iguratimod group before treatment, after 4 weeks of treatment, and after 8 weeks of treatment were (6.28 ± 1.41), (3.22 ± 0.97), and (2.35 ± 0.70) points, respectively. ^*∗*^The remarkable differences in VAS scores between the diclofenac sodium group and the celecoxib group after 4 weeks and 8 weeks of treatment from left to right (*t* = 4.430 and 3.211, *P* < 0.05);  ^*∗∗*^the remarkable differences in VAS scores between the diclofenac sodium group and the iguratimod group after 4 weeks and 8 weeks of treatment from left to right (*t* = 10.652 and 11.549, *P* < 0.05); and  ^*∗∗*^the remarkable differences in VAS scores between the celecoxib group and the iguratimod group after 4 weeks and 8 weeks of treatment from left to right (*t* = 6.156 and 6.746, *P* < 0.05).

**Figure 2:** Comparison of WOMAC scores. The abscissa indicated before treatment and after treatment, and the ordinate indicated the WOMAC score (points). The WOMAC scores in the diclofenac sodium group before treatment and after treatment were (49.16 ± 5.21) and (44.51 ± 4.20) points, respectively. The WOMAC scores in the celecoxib group before treatment and after treatment were (48.79 ± 5.28) and (35.47 ± 3.60) points, respectively. The WOMAC scores in the iguratimod group before treatment and after treatment were (48.85 ± 5.25) and (23.54 ± 4.31) points, respectively.  ^*∗*^The remarkable differences in the WOMAC scores between the diclofenac sodium group and the celecoxib group and between the diclofenac sodium group and the iguratimod group from top to bottom (*t* = 10.336 and 20.038, *P* < 0.001);  ^*∗∗*^the remarkable difference in the WOMAC scores between the celecoxib group and the iguratimod group (*t* = 13.436, *P* < 0.001).

**Table 1:** Comparison of general data (*n* = 40).

Observed indexes	Diclofenac sodium group	Celecoxib group	Iguratimod group	*P*
Age (years)	62.45 ± 3.57	62.78 ± 3.40	62.31 ± 3.62	<0.005
Course of disease (years)	1.85 ± 0.46	1.88 ± 0.44	1.89 ± 0.50	<0.005
BMI (kg/m^2^)	23.71 ± 2.28	23.84 ± 2.30	23.69 ± 2.32	<0.005
*Sex*				<0.005
Male	27 (67.5)	24 (60)	26 (65)	
Female	13 (32.5)	16 (40)	14 (35)	
*Focus of infection*				<0.005
Single knee	31 (77.5)	28 (70)	30 (75)	
Both knees	9 (22.5)	12 (30)	10 (25)	
*K-L classification*				<0.005
Grade I	14 (35)	15 (37.5)	13 (32.5)	
Grade II	26 (65)	25 (62.5)	27 (67.5)	
*Educational level*				<0.005
Under junior middle school	22 (55)	24 (60)	25 (62.5)	
Junior middle school and above	18 (45)	16 (40)	15 (37.5)	

K-L classification represented the classification of the severity of knee osteoarthritis according to Kellgren–Lawrence grading system.

**Table 2:** Comparison of inflammatory factor levels.

Group	IL-6 (ng/mg)	TNF-*α* (pg/mg)	Hs-CRP (mg/L)
Diclofenac sodium group	24.68 ± 4.80	55.18 ± 3.26	3.45 ± 1.20
Celecoxib group	15.22 ± 3.16 ^*∗*^	36.71 ± 4.12 ^*∗*^	3.06 ± 1.04 ^*∗*^
Iguratimod group	10.35 ± 2.47 ^*∗*^^#^	25.61 ± 3.23 ^*∗*^^#^	2.08 ± 0.95 ^*∗*^^#^

*∗*Statistically significant difference compared with the diclofenac sodium group (*P* < 0.05); ^#^statistically significant difference compared with the celecoxib group (*P* < 0.05).

**Table 3:** Comparison of Lysholm scores.

Group	n	Before treatment	After 4 weeks of treatment	After 8 weeks of treatment
Diclofenac sodium group	40	62.53 ± 4.51	67.85 ± 3.87	70.83 ± 2.56
Celecoxib group	40	63.14 ± 3.86 ^*∗*^	75.29 ± 4.01 ^*∗*^	79.69 ± 3.17 ^*∗*^
Iguratimod group	40	62.82 ± 4.49 ^*∗*^^#^	81.06 ± 3.25 ^*∗*^^#^	88.46 ± 3.75 ^*∗*^^#^

*∗*Statistically significant difference compared with the diclofenac sodium group (*P* < 0.05); ^#^statistically significant difference compared with the celecoxib group (*P* < 0.05).

## Data Availability

The data used to support the findings of this study are available from the corresponding author upon reasonable request.
